# Effect of ERAS Combined with Comfortable Nursing on Quality of Life and Complications in Femoral Neck Fractures of the Aged People

This article has been retracted.

**DOI:** 10.1155/2021/8753076

**Published:** 2021-11-03

**Authors:** Hu Ping, Xu Ling, Yiwei Xue, Fanghui Dong

**Affiliations:** ^1^Department of Orthopaedics, Sixth People's Hospital Affiliated to Shanghai Jiaotong University, Shanghai 200233, China; ^2^Department of Nursing, Shanghai Jiao Tong University Affiliated Sixth People's Hospital, Shanghai 200233, China

## Abstract

**Objective:**

To explore the effect of enhanced recovery after surgery (ERAS) combined with comfortable nursing on the quality of life and complications of elderly patients with femoral neck fracture (FNF).

**Methods:**

From May 2019 to May 2020, 80 senile FNF patients who admitted to our hospital were treated by total hip arthroplasty (THA). All patients were randomly divided upon admission into a control group (CG) with usual care and a study group (RG) with ERAS combined with comfort care of 40 patients each. The postoperative efficacy was assessed by Harris score of hip joint function, and the psychology was evaluated by self-rating anxiety scale (SAS). The SF-36 score of quality of life, the time of catheter removal, the time of getting out of bed, the hospital stays, the satisfaction of nursing, and the Barthel score of self-care ability were compared between the two groups before and after nursing, and the incidence of postoperative complications was also evaluated.

**Results:**

Compared with the CG, the SF-36 score of quality of life and Barthel score of self-care ability in the RG were dramatically higher, while the SAS score of anxiety was dramatically lower. Besides, the time of catheter removal, the time of getting out of bed, and the hospital stays in the RG were dramatically lower (*P* < 0.05). Furthermore, the nursing satisfaction and postoperative efficacy of patients in the RG were obviously higher (both *P* < 0.05), while the incidence of complications in the RG was obviously lower (*P* < 0.05).

**Conclusion:**

ERAS combined with comfortable nursing can improve the hip joint function, quality of life, and self-care ability scores of senile FNF patients; relieve the anxiety in patients; and reduce the incidence of postoperative complications, which is valuable to be applied extensively.

## 1. Introduction

In the context of accelerated global aging, China's elderly population is increasing, and elderly patients are a special group. With age, the functions of various tissues and organs of the elderly organism gradually deteriorate, often combined with a variety of medical diseases such as respiratory system, cardiovascular system, and endocrine system [1]. Femoral neck fractures (FNF) are fractures that occur below the head of the femur and above the base of the femoral neck as a result of direct or indirect violence and are a common clinical type of fracture [2]. Fractures of the neck of the femur can occur in older people as a result of slight external forces due to osteoporosis and increased brittleness of the bone in old age, making it the most common condition in older people with a high mortality and disability rate [3]. Total hip arthroplasty (THA) has become a familiar diagnosis and treatment method for orthopedic joint diseases, especially total hip and knee joint replacement [4]. However, due to the physiological particularity of the elderly, the functional recovery of the bones of patients after fracture is often poor [5]. Statistics show that the elderly are prone to infection, deep vein thrombosis (DVT), pulmonary embolism, joint stiffness, and other complications after fracture [6, 7]. Thus, to find an effective rehabilitation and nursing program is a vital task to improve hip joint dysfunction and reduce complications in elderly patients.

The concept of enhanced recovery after surgery (ERAS) first appeared in 1997, which was put forward by Danish scholar Kehlet [8]. With continuous improvement, ERAS has gradually developed into a multidisciplinary team method. More studies [9, 10] have shown that early intervention using the ERAS concept can reduce the occurrence of postoperative complications, reduce the physical and psychological trauma of patients, shorten the length of hospital stay, and accelerate their postoperative recovery. Currently, the ERAS concept is widely used in the care of patients in many departments such as orthopaedics, neurosurgery, and urology and has achieved good results. Comfortable nursing is a new nursing mode, which follows the people-oriented concept and emphasizes patient-centered care; nurses start nursing on the basis of fully understanding patients' needs, which can make them feel respected and cared, thus cooperating with treatment at a higher degree [11, 12]. But it has not been reported whether comfortable nursing is effective in senile FNF patients after THA.

The main purpose of this study is to explore the effect of ERAS combined with comfort nursing on the quality of life and complications of senile FNF patients, so as to provide data support for rehabilitation and nursing treatment.

## 2. Methods and Data

### 2.1. Clinical Data

The clinical data of 80 elderly FNF patients admitted to our hospital from May 2019 to May 2020 were collected, and all patients were assessed and decided to receive THA treatment. Upon admission, all patients were numbered 1 to 80 according to the order of admission and were divided into 40 cases each in the control group (CG) with usual care and the study group (RG) with ERAS combined with comfort care according to the random number table method. This study was approved by the Medical Ethics Committee of our hospital.

### 2.2. Inclusion and Exclusion Criteria

Inclusion criteria: (1) all FNF patients confirmed by CT examination and meeting the indications of THA were operated by the same group of physicians; (2) all of them were ≥60 years old; (3) American Association of Anesthesiologists (ASA) was grades I-II; (4) both family members and patients were informed, and they signed an informed consent form.

Exclusion criteria: (1) the patients had a FNF history and had undergone THA; (2) those with severe chronic systemic diseases; (3) those who were complicated with mental illness and could not cooperate with the treatment; (4) those with other joint dysfunction; (5) those who were complicated with malignancies.

### 2.3. Nursing Plans

The CG was treated by routine nursing, and the specific scheme was as follows: after the patients were admitted to hospital, the primary nurse informs their admission education, psychological nursing, and operation notice. They were fasted for 12 h before operation, deprived of water for 10 h, and given 500 mL enema with normal saline at 20:00 before operation. The operating room temperature was maintained at 24°C, and the infusion and flushing fluid were not specially treated. Drainage tube and urinary catheter were inserted into incision during operation. Liquid diet was given 6 h after anesthesia. The drainage tube was removed on 1-2 days after operation, and the catheter was pulled out after the patients got out of bed or the analgesic pump was removed. According to the pain circumstances, the patients took parecoxi-sodium intramuscular or intravenous, and their rehabilitation was evaluated and rehabilitation exercise was properly performed. Patients can be discharged after removal of stitches or at the request of their families.

The RG adopted ERAS combined with comfortable nursing, which was divided into preoperative, intraoperative, and postoperative nursing. More specifically, the department director, head nurse, doctor in charge of the bed, and primary nurse jointly worked out the rehabilitation process and nursing scheme, while anesthesiologists and nurses worked out the preoperative visit and intraoperative optimization plan. Before operation, the patients were placed in a quiet and comfortable unit ward, and their physical conditions were comprehensively evaluated; the basic diseases were actively treated through department consultation, and the preoperative preparation was done as soon as possible. Psychological nursing: aiming at the patients' psychology, the nursing staff should calm their emotions; explain the relevant knowledge, precautions, postoperative complications, and treatment methods of radiotherapy; eliminate their doubts and fears; relieve the preoperative anxiety and depression symptoms; and reduce the surgical stress response. Intestinal preparation: the nursing staff should pay attention to preoperative fasting and glucose load, patients with diabetes or impaired glucose tolerance should be taken routine fasting measures. Patients with no history of diabetes and impaired glucose tolerance should take 500 mL of carbohydrate solution orally 3 h before operation. During operation, the temperature of the operating room was adjusted to 24°C by the nurse anesthetist 1 h before operation, and the infusion and flushing fluids were heated to 37°C by the incubator. During the transfer from the operating room to the ward, quilts were covered to keep them warm. Besides, the nurses should strictly stop bleeding and prevent reinfusion of autologous blood. No drainage tube was built in incision under special circumstances. After anesthesia, indwelling catheter was given and removed on the first day after operation. Hot water was given 2 h after operation, and liquid diet was given 4 h after operation. Patients with massive bleeding were given subcutaneous injection of erythropoietin or oral ferrous succinate tablets. In the analgesia mode, patients were given preemptive analgesia and multimode analgesia. After that, patients were given patient-controlled analgesia pump and lofenac sustained-release tablets to relieve pain after operation, so as to reduce their discomfort. Rehabilitation training: patients need to carry out rehabilitation exercise as soon as possible, and the doctor in charge of the bed should make a personalized training plan according to their condition. After the patient was awake from postoperative anaesthesia, joint activity training was performed, and abduction of affected limb and hip flexion and knee flexion training were finished in bed. Discharge guidance: the nurses should explain the discharge precautions and the time of outpatient reexamination to patients and their families when they are discharged from the hospital. Also, they should keep abreast of patients' condition through WeChat. Patients were told to take antiosteoporosis drugs and prevent falls. Two groups of patients were nursed under the same nursing team. Homogeneous treatment, examination, and nursing were the first operation on the same day.

### 2.4. Outcome Measures

Scale evaluation: the Harris score was used to assess the patient's hip function before and after the intervention. The score was mainly used to assess the patient's pain, daily function, and physical examination. A short form (SF-36) health survey was used to examine the patients' quality of life after the intervention. The SF-36 scale consists of eight dimensions, each with a score range of 0–100, and the scores of each item in the eight dimensions were counted and converted into standard scores: conversion score = (original score − lowest possible score)/(highest available score − lowest score) × 100%, and the sum of the standard scores of each dimension was the total SF-36 score, with higher scores indicating better quality of life. A modified Barthel Index was used to assess the patient's ability to care for themselves after the intervention, with scores ranging from 0 to 100, the higher the score, the better the patient's ability to perform daily activities. The anxiety self-assessment scale (SAS) was used to assess the patients' psychological state after the intervention. The scale was scored as 50, with a score below 50 indicating no anxiety and a higher score indicating more severe anxiety. A hospital-made satisfaction scale was used to assess the satisfaction level of the two groups, with a total score of 100, ≥90 was very satisfied, ≥70–<90 was basically satisfied, and <70 was unsatisfactory. Satisfaction rate = ((very satisfied + basically satisfied)/total cases) × 100%.

Assessment of efficacy: the efficacy of the treatment was assessed using the Harris scale, with reference indicators including functional recovery, postoperative pain, deformity, and range of motion. The reference indicators included functional recovery, postoperative pain, deformity, and range of motion. A score of 90–100 was considered excellent, a score of 82–89 was considered good, a score of 70–79 was considered moderate, and a score of 70 or less was considered poor.

The time of catheter removal, the time of getting out of bed, the length of hospital stay, and the cost of hospitalization were counted in both groups. The occurrence of postoperative I complications such as pulmonary embolism, infection, joint stiffness, and deep vein thrombosis in the lower limbs was recorded.

### 2.5. Statistical Analysis

SPSS21.0 software package was used for statistical analysis, and GraphPad Prism 8.0 was used for drawing. The measurement data were expressed by mean ± standard deviation (mean ± SD); the comparison method between groups was independent samples *t-*test, while paired *t*-test was used to assess the data within the group. The counting data were expressed by number of cases and percentage (*n*, %), and the comparison method between groups was *χ*^2^ test. A *P* value of <0.05 was a statistical difference.

## 3. Results

### 3.1. Comparison of General Data

The general data of both groups of patients revealed that there was no statistical difference in age, gender, BMI, past medical history, smoking history, and ASA grading (*P* > 0.05, Table 1).

### 3.2. Efficacy Evaluation

We evaluated the clinical efficacy of patients after 6 months of treatment. It was found that the clinical efficacy of patients in the CG was dramatically lower than that of those in the RG, and there was a statistical difference (*P* < 0.05, Tables 2 and Table 3).

### 3.3. Comparison of Patients' Quality of Life, Self-Care Ability, and Anxiety

The quality of life, self-care ability, and anxiety of patients in both groups after treatment demonstrated that the quality of life and self-care ability of patients in the CG were dramatically lower than those in the RG (*P* < 0.05, Figure 1).

Comparison of postoperative conditions such as time of catheter removal, time of getting out of bed, length of stay, and hospitalization expenses between the two groups is done.

This study also compared the time of catheter removal, the time of getting out of bed, the length of stay, and the hospitalization expenses of patients. It was discovered that the first three in the CG were dramatically higher than those in the RG, with statistical difference (*P* < 0.05). Furthermore, further comparative analysis manifested that the hospitalization expenses of patients in the CG were dramatically higher than those in the RG, and there was a statistical difference (Figure 2, *P* < 0.05).

### 3.4. Comparison of Nursing Satisfaction

In this study, patients were graded for their satisfaction with the nursing process. From the comparison, it was found that the nursing satisfaction of patients in the CG was dramatically lower than that in the RG (*P* < 0.05). Moreover, the satisfaction rate of patients in the CG was dramatically lower, with statistical difference (*P* < 0.05, Table 4).

### 3.5. Incidence of Complications

At the end of the study, we made statistics on postoperative complications. It is concluded that there was no difference in intestinal reaction, infection, and incidence of femoral head necrosis between both groups (*P* > 0.05). But the incidence of DVT in the CG was dramatically higher than that in the RG, with statistical difference (*P* < 0.05, Table 5).

## 4. Discussion

Recently, with the sharp increase of aging population, the morbidity of FNF in middle-aged and elderly people is increasing, which has a serious impact on patients' daily life [13, 14]. FNF is a common fracture type in the elderly [15]. Once suffering from it, the ability of blood circulation supply becomes poor, and patients with conservative treatment need to stay in bed for a long time, which is prone to complications such as falling pneumonia and venous thrombosis [16].

The traditional treatment method is to drag the patient or break the affected limb, which takes a long time and is prone to pneumonia, venous thrombosis, and other complications; seriously, it may bring about death [17, 18]. ERAS, as a new and scientific rehabilitation model, is an advanced surgical perioperative treatment theory in Europe, which is widely used in general surgery and obstetrics and gynecology perioperative period [19]. Its idea is based on evidence-based medicine, through optimizing various perioperative treatment measures, combined with many independent disciplines, such as surgery, rehabilitation, anesthesiology, nursing, and psychology; on the premise of taking patients as the center, it achieves the purpose of promoting patients' rehabilitation through coordination and cooperation, and its value in clinical treatment has been confirmed by many reports abroad [20, 21]. Comfortable nursing is a holistic and creative nursing mode, which aims to make patients feel comfortable both physically and psychologically [22]. In this study, we intervened in senile FNF through ERAS combined with comfortable nursing. We can conclude through comparative research that the clinical efficacy of patients in the RG was dramatically higher than that in the CG after joint intervention. Afterwards, patients' quality of life and self-care ability were improved, and their anxiety was eliminated. This is mainly because ERAS combined with comfort nursing intervention can alleviate patients' anxiety through proper preoperative health education and effective psychological nursing [23]. According to the situation of each patient, targeted psychological counseling is carried out, and the surgical plan and rehabilitation measures are explained in detail, so that the patients and their families can actively cooperate with the operation and get through the perioperative period safely [24].

Perioperative pain is the main cause of stress response and also the main reason for preventing patients from rehabilitation training as soon as possible. Preemptive analgesia can reduce perioperative stress response, postoperative pain, and the risk of postoperative complications [25, 26]. Excessive fluid replacement during perioperative period can affect the rehabilitation process of patients after operation, and unlimited fluid replacement after operation will also prolong the hospital stay. In this study, we reduced fluid replacement for patients and relived central nervous system complications and cognitive impairment by using preemptive analgesia, thus shortening the time for catheter removal, time of getting out of bed, and length of stay and hospitalization expenses after operation [23]. The meta-analysis of Elsarrag et al. [27] told that ERAS dramatically shortened the length of stay and readmission rate after spinal surgery; it also reduces postoperative pain, saves hospitalization expenses, and improves the incidence of adverse reactions, which is consistent with our research results.

DVT is a familiar complication of THA [28]. It is reported that the incidence rate is as high as 50%, and about 80% of DVT patients have no obvious clinical symptoms. Once the embolus of DVT patients falls off, it will lead to pulmonary embolism and even endangers life [29, 30]. In the present study, we found a reduction in the incidence of lower limb DVT in RG compared to CG after the combined intervention. This denotes that combined intervention can reduce the DVT formation of lower limbs. This is mainly due to the fact that negative pressure drainage tube and catheter are not retained as far as possible in the ERAS scheme, and if they must be retained, they should be removed as soon as possible after operation, which can reduce the complications caused by pipelines and facilitate patients to get out of bed early. Based on patients' physical condition, we developed targeted rehabilitation training, which accelerated their postoperative recovery, thereby reducing the DVT formation of lower limbs.

We have confirmed the clinical value of intensive rehabilitation combined with comfortable nursing for senile FNF patients through analysis. Nevertheless, this study still has some limitations. First of all, we did not follow-up the patients for a long time, and the longest was only one year. It is not clear whether the two different schemes have an impact on the postoperative survival of patients. Furthermore, our sample is small, so it is impossible to analyze the risk factors of DVT of lower limbs. Hence, we hope to collect more samples in future studies and make long-term follow-up and analysis to complete our data.

To sum up, ERAS combined with comfortable nursing can improve the quality of life of senile FNF patients, relieve their negative emotion, and reduce the incidence of DVT, which deserves to be generalized.

## Figures and Tables

**Figure 1:** Comparison of quality of life, self-care ability, and anxiety of patients. (a) Comparison of SF-36 score of quality of life. (b) Comparison of Barthel score of self-care ability. (c) Comparison of anxiety SAS score.  ^*∗*^*P* < 0.05;  ^*∗∗*^*P* < 0.01.

**Figure 2:** Comparison of time of catheter removal, time of getting out of bed, length of stay, and hospitalization expenses. (a) Time of catheter removal after operation. (b) Time of getting out of bed after operation. (c) Postoperative hospital stays. (d) Comparison of hospitalization expenses of patients.  ^*∗∗∗*^*P* < 0.001.

**Table 1:** Comparison of general data.

Factor		Control group (*n* = 40)	Research group (*n* = 40)	*P* value
Age (*n*)				0.159
	≥65 years old	29	23	
	60∼65 years old	11	17	
Gender (*n*)				0.259
	Man	25	20	
	Woman	15	20	
BMI (*n*)				0.648
	≥22 kg/m^2^	17	15	
	˂22 kg/m^2^	23	25	
Past medical history (*n*)				
	Diabetes	8	12	0.302
	Hypertension	13	10	0.458
History of smoking (*n*)				0.119
	Yes	27	20	
	No	13	20	
ASA grading (*n*)				0.651
	Grade I	18	16	
	Grade II	22	24	

**Table 2:** Harris score of hip function (mean ± SD, scores).

Grouping	Before nursing	After nursing
CG (*n* = 40)	66.79 ± 5.61	80.57 ± 6.35
RG (*n* = 40)	66.81 ± 5.59	88.69 ± 7.01
*t* value	0.016	5.430
*P* value	0.987	≤0.01

**Table 3:** Efficacy evaluation (*n*, %).

Grouping	Excellent	Good	Moderate	Bad	Excellent and good rate
CG (*n* = 40)	6	20	9	5	26 (41.27)
RG (*n* = 40)	14	23	2	1	37 (58.73)
*Z*/*χ*^2^ value	−3.942				9.038
*P* value	<0.001				0.003

**Table 4:** Nursing satisfaction (*n*, %).

Grouping	Very satisfied	Basically satisfied	Dissatisfied	Satisfaction rate
CG (*n* = 40)	25	11	4	36 (90.00)
RG (*n* = 40)	10	16	14	26 (65.00)
Z/*χ*^2^ value	−3.058			7.168
*P* value	0.002			0.007

**Table 5:** Incidence of complications (*n*).

Grouping	Pulmonary embolism	Infection	Joint stiffness	Deep venous thrombosis of lower limbs
CG (*n* = 40)	3	3	2	6
RG (*n* = 40)	2	1	1	1
*χ* ^2^ value	0.213	1.053	0.321	3.914
*P* value	0.644	0.305	0.571	0.048

## Data Availability

The data are available from the corresponding author upon request.
